# Grape Seed Proanthocyanidins Inhibit the Invasiveness of Human HNSCC Cells by Targeting EGFR and Reversing the Epithelial-To-Mesenchymal Transition

**DOI:** 10.1371/journal.pone.0031093

**Published:** 2012-01-27

**Authors:** Qian Sun, Ram Prasad, Eben Rosenthal, Santosh K. Katiyar

**Affiliations:** 1 Birmingham Veterans Affairs Medical Center, Birmingham, Alabama, United States of America; 2 Department of Dermatology, University of Alabama at Birmingham, Alabama, United States of America; 3 Department of Surgery-Otolaryngology, University of Alabama at Birmingham, Alabama, United States of America; 4 Comprehensive Cancer Center, University of Alabama at Birmingham, Birmingham, Alabama, United States of America; University of Saarland Medical School, Germany

## Abstract

Head and neck squamous cell carcinoma (HNSCC) is responsible for approximately 20,000 deaths per year in the United States. Most of the deaths are due to the metastases. To develop more effective strategies for the prevention of metastasis of HNSCC cells, we have determined the effect of grape seed proanthocyanidins (GSPs) on the invasive potential of HNSCC cell and the mechanisms underlying these effects using OSC19 cells as an *in vitro* model. Using cell invasion assays, we established that treatment of the OSC19 cells with GSPs resulted in a dose-dependent inhibition of cell invasion. EGFR is over-expressed in 90% of HNSCCs and the EGFR inhibitors, erlotinib and gefitinib, are being explored as therapies for this disease. We found that GSPs treatment reduced the levels of expression of EGFR in the OSC19 cells as well as reducing the activation of NF-κB/p65, a downstream target of EGFR, and the expression of NF-κB-responsive proteins. GSPs treatment also reduced the activity of ERK1/2, an upstream regulator of NF-κB and treatment of the cells with caffeic acid phenethyl ester, an inhibitor of NF-κB, inhibited cell invasion. Overexpression of EGFR and high NF-κB activity play a key role in the epithelial-to-mesenchymal transition, which is of critical importance in the processes underlying metastasis, and we found treatment with GSPs enhanced the levels of epithelial (E-cadherin, cytokeratins and desmoglein-2) and reduced the levels of mesenchymal (vimentin, fibronectin, N-cadherin and Slug) biomarkers in the OSC19 cells. These results indicate that GSPs have the ability to inhibit HNSCC cell invasion, and do so by targeting the expression of EGFR and activation of NF-κB as well as inhibiting the epithelial-to-mesenchymal transition.

## Introduction

Squamous cell carcinoma of the head and neck (HNSCC) is the sixth most commonly occurring malignancy world-wide. It is responsible for approximately 20,000 deaths and affects more than 40,000 people in the United States annually [1], [2]. HNSCCs exhibit aggressive behavior with a high incidence of secondary primaries in the head and neck (5–7% per year) together with a high incidence of distant metastases. This potent metastatic capacity is associated closely with the high mortality rate. Advances in surgical and medical therapies for HNSCC have resulted in only a modest improvement in the mortality rate, which has remained at approximately 50% for the last three decades [3]–[6]. Currently available therapies including conventional chemotherapy and surgical resection are often associated with severe morbidity due to the involvement of vital structures of the head and neck, side effects and therapeutic resistance. Therefore, elucidation of the molecular pathways essential for metastasis and identification of approaches that minimize the invasive and metastatic behaviors of cancer cells is of high priority in the treatment of patients with HNSCC and in chemoprevention.

Naturally occurring bioactive dietary phytochemicals that are non-toxic and devoid of major side effects are candidates for the prevention of recurrence or metastasis of cancer cells. Such agents can be utilized as complementary and alternative medicine and/or as adjuvant therapy for conventional cytotoxic therapies. The seeds of grapes (*Vitis vinifera* L.) are a rich source of proanthocyanidins and these grape seed proanthocyanidins (GSPs) are promising bioactive phytochemicals that have shown anti-carcinogenic effects in some tumor models with no apparent signs of toxicity in these animal models [7]–[9]. In spite of the anti-carcinogenic effects of GSPs [7], their chemotherapeutic effects on the invasive potential of HNSCC cells have not been assessed.

Epidermal growth factor receptor (EGFR) appears to play a critical role in HNSCC. It is overexpressed in almost all HNSCC tumors (>90%) and its overexpression is associated with poor prognosis [10]–[12]. It has been reported that small molecule inhibitors of EGFR, such as erlotinib and gefitinib, can prevent the growth and progression of HNSCCs [13]. A downstream target of EGFR, the transcription factor nuclear factor-kappaB (NF-κB), also has been shown to be essential for metastasis in models of cancer progression [14]. The overexpression of EGFR, enhanced EGFR-associated signaling, and enhanced NF-κB activity have all been linked to the epithelial-to-mesenchymal transition (EMT). During EMT, cancer cells lose expression of proteins that promote cell-cell contact, such as E-cadherin, and acquire mesenchymal markers, such as vimentin, fibronectin and N-cadherin, that promote tumor progression, cell invasion and metastasis [15], [16]. In the present communication, we explored the chemotherapeutic effects of GSPs on the invasive potential of human HNSCC cells and ascertained whether EGFR and its associated pathways are involved in this process. Comparison of the invasive potential of several different HNSCC cell lines derived from different sub-sites indicated that the OSC19 cell line exhibited the greatest invasive potential and this cell line was used in all subsequent studies. We report that GSPs inhibit the invasive potential of the OSC19 HNSCC cells through inhibition or reversal of EMT and that this GSPs-induced inhibition is accomplished through a process that involves a reduction in the levels of EGFR expression, inactivation of NF-κB and inactivation of Erk1/2.

## Materials and Methods

### Source of the grape seed proanthocyanidins

The GSPs preparation was received from the Kikkoman Company, Noda, Japan (no financial conflict of interest) and used throughout the study. Quality control of the GSPs preparation is maintained by the company on lot-to-lot basis. The GSPs preparation contains approximately 89% proanthocyanidins, with dimers (6.6%), trimers (5.0%), tetramers (2.9%) and oligomers (74.8%), as described earlier [7]–[9]. The product is stable for at least two years when refrigerated at 4°C.

### Chemicals, reagents and antibodies

Boyden Chambers and polycarbonate membranes (8 µm pore size) for cell migration/invasion assays were obtained from Neuroprobe, Inc. (Gaithersburg, MD). The antibodies specific for N-cadherin, keratin 8, keratin 18, fibronectin, EGFR, ERK1/2, cyclooxygenase-2 (COX-2), matrix metalloproteinase (MMP)-2, MMP-9, inducible nitric oxide synthase (iNOS) and β-actin were obtained from Santa Cruz Biotechnology (Santa Cruz, CA), while antibodies for vimentin, E-cadherin, Slug, NF-κB, IκB kinase α (IKKα), IκBα and vascular endothelial growth factor (VEGF) were purchased from Cell Signaling Technology (Beverly, MA), while desmoglein 2 was obtained from Abcam (Cambridge, MA). The appropriate secondary antibodies conjugated with horseradish peroxidase were procured from Invitrogen (Carlsband, CA). UO126, an inhibitor of the mitogen-activated/extracellular protein-regulated kinase (MEK), was purchased from Sigma Chemical Co. (St. Louis, MO). Erlotinib was procured from Santa Cruz Biotechnology and gefitinib from Toronto Research Chemicals, Inc. (North York, ON, Canada).

### Cell lines and cell culture conditions

HNSCC cell lines derived from the oral cavity (UM-SCC1), larynx (UM-SCC5), pharynx (FaDu) and tongue (OSC19) were obtained from Dr. Rosenthal (University of Alabama at Birmingham, Birmingham, AL). The OSC19 cell line was developed from tumor cells that had metastasized to the lymph node from an HNSCC of the tongue. The cells were cultured as monolayers in DMEM supplemented with 10% heat-inactivated fetal bovine serum and 100 µg/mL penicillin-streptomycin (Invitrogen), and kept in a humidified atmosphere of 5% CO_2_ at 37°C. Cells were seeded at a density of 1×10^6^ cells per culture dish and allowed to attach for 24 h, at which time they were sub-confluent, before treatment with GSPs or other agents. The GSPs, erlotinib or gefitinib were dissolved in a small amount of dimethylsulfoxide (DMSO), which was added to the complete cell culture medium. The maximum concentration of DMSO in media was 0.1% (v/v). Cells treated with DMSO only served as a vehicle control.

### Cell proliferation assay

The effect of GSPs on the viability or cell proliferation of normal human bronchial epithelial cells or human HNSCC cells was determined by 3-(4,5-dimethylthiazol-2-yl)-2,5-diphenyltetrazolium bromide assay (Sigma) or MTT assay, as previously described [17]. A total of 1×10^4^ cells per well in 200 µL complete medium were seeded in a 96-well plate and treated with varying concentrations of GSPs for 48 h. The cells were treated with 50 µL of 5 mg/mL MTT and the resulting formazan crystals were dissolved in dimethylsulfoxide (200 µL). Absorbance was recorded at 540 nm with a reference at 650 nm serving as the blank. The effect of GSPs on cell viability was assessed as percent cell viability compared to vehicle-treated control cells, which were arbitrarily assigned 100% viability. All treatment concentrations were repeated in six wells.

### Cell death assay

The trypan blue dye exclusion assay was used to determine the cytotoxic effect of GSPs on the cells. Briefly, 5×10^4^ cells were cultured into each well of a six-well culture plates. After overnight incubation, the cells were treated with varying concentrations of GSPs (0, 10, 20, 40 µg/mL) for 48 h. Thereafter cells were harvested, treated with 0.25% trypan blue dye and the cells that had taken up the dye were counted under a microscope using a hemocytometer, as detailed previously [17]. The cytotoxic effects of GSPs are expressed as the mean±SD percentage of dead cells in each treatment group from three repeated experiments.

### Cell invasion assay

The invasion capacity of HNSCC cells was determined *in vitro* using Boyden Chambers (Gaithersburg, MD). In this assay, the two chambers were separated with Matrigel-coated Millipore membranes (6.5 mm diameter filters, 8 µM pore size), as detailed previously [18], [19]. Briefly, cells (1.5×10^4^ cells/100 µL serum-reduced [0.5% FBS] medium) were placed in the upper chamber of the Boyden chambers and the test agents were added alone, or in combination, to the upper chamber (200 µL). The lower chamber contained the medium alone (150 µL). The chambers were assembled and kept in a cell culture incubator for the specified periods of time. After incubation, cells from the upper surface of the Millipore membranes were removed with gentle swabbing and the cells on the lower surface of membranes were fixed and stained with crystal violet. The membranes were examined microscopically and cellular invasion was determined by counting the migrating/invasive cells on each membrane in at least 4–5 randomly selected fields using an Olympus BX41 microscope. Representative photomicrographs were obtained using a Qcolor5 digital camera system fitted to an Olympus BX41 microscope. Each experiment was repeated three times and the resultant cell invasion data are presented in terms of the mean number of invasive or migrating cells±SD/microscopic field (magnification, ×10) from three independent experiments.

### Assay for NF-κB/p65 activity

The NF-κB Trans^AM^ Activity Assay Kit (Active Motif, Carlsbad, CA) was used for quantitative analysis of NF-κB/p65 activity following the manufacturer's protocol. For this purpose, the nuclear extracts of cells from various treatment groups were prepared using the Nuclear Extraction Kit (Active Motif, Carlsbad, CA) following the manufacturer's instructions and as described previously [20]. Briefly, this assay kit is an ELISA-based kit to detect and quantify NF-κB activation. By using an antibody that is directed against the NF-κB/p65 subunit, the activated NF-κB/p65 subunit bound to the oligonucleotide is detected. Addition of a secondary antibody conjugated to horseradish peroxidase provides sensitive colorimetric readout that is easily quantified by spectrophotometer. The manufacturer suggests that this NF-κB/p65 Trans^AM^ activity assay kit is more sensitive than EMSA. Absorbance was recorded at 450 nm using absorbance at 650 nm as the reference. The results are expressed as the percentage of the optical density of the non-GSPs-treated control group.

### Western blot analysis

After incubation of cells for the indicated time periods with or without the treatment of GSPs or other agents, the cells were harvested, washed with cold PBS and lysed with ice-cold lysis buffer supplemented with protease inhibitors, as detailed previously [18], [19]. Cytoplasmic and nuclear protein fractions were prepared separately for the analysis of respective proteins. The purity of cytoplasmic and nuclear fractions was tested. The absence of β-actin in nuclear fraction confirms its purity while absence of Lamin B or Histone H3 proteins in cytoplasmic fraction suggests that this fraction is free from nuclear fraction. The purity was confirmed using western blot analysis. Proteins (30–50 µg) were resolved on 10% Tris-Glycine gels and transferred onto a nitrocellulose membrane. After blocking the non-specific binding sites, the membrane was incubated with the primary antibody at 4°C overnight. The membrane was then incubated with the appropriate peroxidase-conjugated secondary antibody and the specific-protein bands were visualized using the enhanced chemiluminescence reagents. The equal loading of protein samples on the gel was verified after stripping and re-probing of the membrane with anti-β-actin antibody. Representative blots are shown from three independent experiments.

### Statistical analysis

For statistical analysis of cell invasion assays, the control, gefitinib, erlotinib or GSPs treatment groups or combined-treatment groups separately were compared using one-way analysis of variance (ANOVA) followed by the *post hoc* Dunn's test using GraphPad Prism version 4.00 for Windows software (GraphPad Software, San Diego, California. www.graphpad.com.) All quantitative data for cell migration are shown as the mean number of migrating cells±SD/microscopic field from at least three independent experiments. In each case *P*<0.05 was considered statistically significant.

## Results

### Analysis of the invasive potential of human HNSCC cells

First, we assessed the invasion capacity of various HNSCC cell lines that originated from different sub-sites of the head and neck, including the oral cavity (SCC1), larynx (SCC5), pharynx (FaDu) and tongue (OSC19) using a modified Boyden chamber assay. Incubation of the HNSCC cells for 48 h resulted in a greater number of invasive cells than incubation for 24 h. Representative photographs of crystal violet-stained membranes are shown in Figure 1A. As shown in Figure 1B, calculation of the cell invasion data in terms of the mean number of invasive cells±SD/microscopic field (magnification, ×10), the invasion capacity of OSC19 cells was found to be greater (380±16 cells/microscopic field) than SCC1 (75±7), SCC5 (38±4) and FaDu (58±5) cells. The invasion capacity of OSC19 cells was significantly higher (*P*<0.001) than that of SCC1, SCC5 and FaDu cells. Under identical conditions, the migration of normal human bronchial epithelial cells was hardly detectable (data not shown). As the invasive potential of OSC19 cells was significantly greater than other HNSCC cell lines tested under the conditions of this assay, the OSC19 cell line was selected for further studies.

**Figure 1:** Analysis of invasive potential of HNSCC cell lines. (**A**) The invasion potential of several human HNSCC cell lines including SCC1 (derived from the oral cavity), SCC5 (derived from the larynx), FaDu (derived from the pharynx) and OSC19 (derived from a lymph-node metastases from the tongue) were assessed using a Boyden chamber cell invasion assay. Equal numbers of cells were loaded and after 48 h incubation, invasive cells were detected on the membrane by staining with crystal violet. (**B**) The invasive cells were counted and the results expressed as the mean number of invasive cells±SD/microscopic field, magnification: ×10. Significantly higher *versus* other cells, ^*^ *P*<0.001.

### GSPs inhibit the invasive potential of OSC19 cells

To determine whether bioactive phytochemicals have the ability to inhibit the invasive potential of HNSCC cells, we used GSPs as a test agent in the *in vitro* cell invasion assay described above. As shown in Figure 2, as compared to non-GSPs-treated control cells, the treatment of cells with GSPs at the concentrations of 10, 20 and 40 µg/mL for 48 h reduced the invasive potential of OSC19 cells in a concentration-dependent manner. The density of the migrating cells on the membrane after staining with crystal violet is shown in Figure 2A, and a summary of the mean numbers of invasive cells±SD/microscopic field is provided in Figure 2B. The cell invasion potential of the OSC19 cells was inhibited by 41–81% (*P*<0.05−0.001) in a concentration-dependent manner after treatment with GSPs. To verify that the inhibition of invasion of OSC19 cells by the GSPs was due to a direct effect on migration ability, and was not due to a reduction in cell viability, a trypan blue assay was performed using cells that were treated identically to those used in the cell invasion assays. Treatment of OSC19 cells with various concentrations of GSPs (0, 10, 20 and 40 µg/mL) for 48 h had no significant effect on cell viability or induction of cell death (data not shown). Similarly, we also checked the toxic effects of GSPs on normal bronchial epithelial cells *in vitro*. These cells were treated with various concentrations of GSPs for 24 and 48 h under identical conditions. As shown in Figure 2C, treatment of cells with GSPs did not reduce significantly the proliferation ability or viability of cells as well as could not induce significant cell death under the experimental conditions used in this study. These data suggest that GSPs are not toxic to normal bronchial epithelial cells.

**Figure 2:** Effect of GSPs on HNSCC cell invasion and EGFR expression. (**A**) OSC19 cells were treated with the indicated concentrations of GSPs for 48 h and the effects on their invasiveness assessed as described in Figure 1. Crystal violet staining of the membranes showed that, as compared to non-GSPs-treated control cells, the GSPs inhibited invasion of cells in a concentration-dependent manner. (**B**) The migratory cells were counted and the results expressed as the mean number of invasive cells±SD/microscopic field, magnification: ×10. The values are reported from three separate experiments. Significant inhibition *versus* non-GSPs-treated control, ^*^ *P*<0.001, ^¶^ *P*<0.01. (**C**) The non-toxic effect of GSPs on normal human bronchial epithelial cells was determined in terms of cell viability and cell death. The data on cell viability are expressed in terms of percent of control cells (non-GSPs-treated) as the mean±SD of 6 replicates. Similarly, the cytotoxic effect of GSPs on normal bronchial epithelial cells was determined using trypan blue dye exclusion assay as described in Materials and Methods and is expressed in terms of percent of dead cells as mean±SD from three experiments. (**D**) Dose-dependent effect of GSPs on EGFR expression in OSC19 cells. The levels of EGFR in whole cell lysates of OSC19 cells treated with different concentrations of GSPs for 48 h were determined using western blot analysis. Representative blots are shown from three independent experiments.

### Treatment of cells with GSPs reduces the level of EGFR expression

As it has been shown that EGFR is overexpressed in over 90% of HNSCC tumors [10]–[12], we determined whether inhibition of cell invasion of OSC19 cells by GSPs is associated with a reduction in the expression of EGFR. For this purpose, whole cell lysates from different treatment groups were analyzed by western blotting. As shown in Figure 2D, treatment of OSC19 cells with GSPs for 48 h resulted in a reduction in the levels of EGFR expression in a concentration-dependent manner as compared to the expression of EGFR in non-GSPs-treated controls. These results suggest that the GSPs-induced reduction in EGFR expression may be associated with an inhibitory effect of the GSPs on the invasive potential of these cells.

### The EGFR inhibitors, erlotinib and gefitinib, inhibit the invasive potential of OSC19 cells

We next examined the effects of the erlotinib, a selective inhibitor of EGFR, and gefitinb, a kinase inhibitor that inhibits EGFR, on the cell invasion potential of the OSC19 cells. For this purpose, cells were incubated with various concentrations of erlotinib (0, 0.1, 1.0 and 10.0 µM) for 48 h in Boyden chambers. As shown in Figure 3A, treatment of the cells with erlotinib resulted in a dose-dependent reduction in the cell invasion capacity of OSC19 cells as reflected by the presence of invasive cells on the membrane compared with non-erlotinib-treated controls. The resultant data on cell invasion was determined in terms of the number of invasive cells/microscopic field±SD at different concentrations of erlotinib and are summarized in Figure 3B. Similar results were obtained when OSC19 cells were treated with gefitinib. Resultant data on cell invasion which are shown in Figure 3C and are summarized in Figure 3D, demonstrated that the treatment of OSC19 cells with gefitinib for 48 h under identical conditions resulted in a dose-dependent inhibition of cell invasion. These results support the concept that the GSPs may act to inhibit the invasion of OSC19 HNSCC cells by targeting the EGFR.

**Figure 3:** Effect of the EGFR inhibitors, gefitinib and erlotinib, on HNSCC cell invasion. (**A**) OSC19 cells were treated with the indicated concentrations of erlotinib, a small molecule inhibitor of EGFR, for 48 h and the effects on invasion assessed as described in Figure 1. Crystal violet staining of the membrane shows that erlotinib inhibited invasion of OSC19 cells in a concentration-dependent manner. (**B**) The invasive cells were counted and the results expressed as the mean number of invasive cells±SD/microscopic field, magnification: ×10. (**C**) Similarly, treatment of OSC19 cells with the indicated concentrations of gefitinib, a small molecule inhibitor of tyrosine kinase activity and, thus, of EGFR, inhibited cell invasion in a dose-dependent manner as indicated by crystal violet staining of the membrane. (**D**) The invasive cells from the experiment described in Figure 3C were counted and the results expressed as the mean number of invasive cells±SD/microscopic field, magnification: ×10. Significant reduction of cell invasion versus untreated control cells, ^¶^ *P*<0.05, ^*^ *P*<0.001.

### GSPs reduce the level and activity of NF-κB/p65 in HNSCC cells: NF-κB is an important mediator of cell invasion

As NF-κB is a down-stream target of EGFR, we assessed whether GSPs affect the levels and activation of NF-κB in OSC19 cells. OSC19 cells were incubated with various concentrations of GSPs (10, 20 and 40 µg/mL) for 48 h, and thereafter the cells were harvested and cytoplasmic and nuclear fractions were prepared for western blot analysis. As shown in Figure 4A, western blot analysis of the nuclear fraction revealed that treatment of cells with GSPs reduced the translocation of NF-κB/p65 into the nucleus in a concentration-dependent manner. The results also indicated that treatment with GSPs resulted in the downregulation of IKKα whereas increases the levels of IκBα, which leads to the inactivation of NF-κB and its translocation to the nucleus. The activity of NF-κB/p65 was significantly reduced in a concentration-dependent manner (30–75%, *P*<0.05, *P*<0.001) after treatment of the cells with GSPs (Figure 4B). Similar results were observed when the OSC19 cells were treated with erlotinib under identical experimental conditions (Figures 4C, 4D). To further assess whether NF-κB has a role in HNSCC cell invasion, OSC19 cells were treated with caffeic acid phenethyl ester (0, 5.0 and 10.0 µg/mL), a potent inhibitor of NF-κB, and cell invasion was determined. As shown in Figure 4E, treatment of OSC19 cells with caffeic acid phenethyl ester resulted in a significant reduction of cell invasion (38% and 64%; *P*<0.05, and *P*<0.001) compared to non-caffeic acid phenethyl ester-treated control cells, and these results are similar to that observed on treatment of the cells with GSPs (Figure 2A, 2B).

**Figure 4:** Effect of GSPs and erlotinib on NF-κB activation in OSC19 cells. (**A**) Treatment of OSC19 cells with GSPs decreases the basal levels of NF-κB/p65 and IKKα while inhibiting the degradation of IκBα. After treatment of cells for 48 h with various concentrations of GSPs the cells were harvested, cytosolic and nuclear fractions were prepared and these were subjected to western blot analysis. Representative blots are shown from three independent experiments with identical observations. (**B**) The activity of NF-κB/p65 in the nuclear fraction of cells after treatment with and without GSPs was measured using an NF-κB/p65-specific activity assay kit, n = 3. Activity of NF-κB/p65 is expressed in terms of percent of the control (non-GSPs-treated) group. Significant decrease versus control: ^¶^ *P*<0.05, ^*^ *P*<0.001. (**C**) Similarly, treatment of OSC19 cells with erlotinib reduced the levels of NF-κB and IKKα. Representative blots are shown from two independent experiments. (**D**) The activity of NF-κB/p65 in the nuclear fraction of cells after treatment with and without erlotinib for 48 h was measured using the NF-κB/p65-specific activity assay kit, n = 2. Activity of NF-κB/p65 is expressed in terms of percent of control (non-erlotinib-treated) group. Significant decrease versus control: ^*^ *P*<0.001. (**E**) Treatment of OSC19 cells with caffeic acid phenethyl ester (CAPE), an inhibitor of NF-κB, for 48 h inhibited cell invasion in a concentration-dependent manner. Data on cell invasion are summarized as the mean number of invasive cells±SD/microscopic field from three independent experiments, magnification: ×10. Significant inhibition *versus* non-CAPE-treated cells, ^*^ *P*<0.001, ^¶^ *P*<0.05. (**F**) GSPs reduce the levels of NF-κB-targeted proteins, such as MMP-2, MMP-9, COX-2, iNOS and VEGF, in OSC19 cells. After treatment of cells with and without GSPs for 48 h, cells were harvested, and cell lysates were subjected to the analysis of the levels of proteins using western blot analysis. Representative blots are shown from three independent experiments.

### GSPs inhibit the expression of NF-κB-targeted proteins in OSC19 cells

As the functional activity of NF-κB is mediated through its targeted proteins, we further determined whether GSPs affect the levels of NF-κB-responsive proteins associated with cancer cell invasion, including MMPs, COX-2, iNOS and VEGF, in HNSCC cells. As shown in Figure 4F, western blot analysis revealed that treatment of OSC19 cells with GSPs resulted in a markedly reduced levels of MMP-2, MMP-9, COX-2, iNOS and VEGF proteins as compared to non-GSPs-treated controls, which is indicated by the visual intensity of the respective bands.

### GSPs as well as MEK inhibitor (UO126) inhibit the phosphorylation of ERK1/2 in OSC19 cells: UO126 reduces the invasive potential of OSC19 cells

Mitogen-activated protein kinases (MAPKs) are down-stream targets of EGFR signaling as well as upstream regulators of NF-κB, and have been implicated in cancer cell metastasis [21]. Therefore, we examined the effect of GSPs on activation of the extracellular-signal regulated kinase (ERK1/2) in HNSCC cells. Western blot analysis revealed that treatment of OSC19 cells with GSPs for 48 h inhibited the phosphorylation of ERK1/2 in a dose-dependent manner, as shown in Figure 5A. Similarly, the treatment of cells with UO126 also inhibited the phosphorylation of ERK1/2 (Figure 5B). We then determined the role of activated ERK1/2 on OSC19 cell invasion. The cell invasion assay revealed that treatment of OSC19 cells with UO126 for 48 h significantly inhibited (68%, *P*<0.001) the invasiveness of cells (Figure 5C, 5D). A summary of data obtained from three independent experiments is shown in Figure 5D.

**Figure 5:** Both GSPs and MEK inhibitor (UO126) inhibit OSC19 cell invasion by reducing activation of ERK1/2. (**A**) GSPs inhibit the activation of ERK1/2 in OSC19 cells in a dose-dependent manner. OSC19 cells were treated with indicated concentrations of GSPs for 48 h, the cells harvested and whole cell lysates subject to western blotting using antibodies specific for total ERK1/2 and phosphorylated ERK1/2. (**B**) Similarly, the treatment of OSC19 cells with UO126, a MEK inhibitor, (80 µM) for 48 h inhibited the activation of ERK1/2 in cells as determined by western blot analysis. Representative blots are shown from three separate experiments. (**C**) OSC19 cells were treated with UO126 (80 µM) for 48 h and cell invasion assessed as described in Figure 1. Crystal violet staining of the membrane indicated that UO126 inhibited the invasive potential of cells as compared to non-UO126-treated control cells. (**D**) The data on cell invasion are summarized and expressed as the mean number of invasive cells±SD/microscopic field, magnification: ×10. Experiments were repeated two times. Significant difference versus control ^*^ *P*<0.001.

### GSPs promote transition of the mesenchymal state to the epithelial state in HNSCC cells

Upregulation of EGFR and activation of downstream targets like ERK1/2 and NF-κB play critical roles in the EMT [15], [16], [21], which has been implicated in cancer cell invasion and metastasis. Therefore, we checked the effect of GSPs on the EMT in OSC19 cells. For this purpose, OSC19 cells were incubated with varying concentrations of GSPs and erlotinib separately for 48 h. Thereafter, cells were harvested and cell lysates were prepared for the analysis of epithelial and mesenchymal biomarkers using western blot analysis. Western blot analyses revealed that GSPs increased the levels of epithelial biomarkers, such as E-cadherin, keratin 8, keratin 18 and desmoglein 2 in OSC19 cells in a dose-dependent manner compared to untreated controls (Figure 6A). In contrast, the levels of mesenchymal biomarkers, such as N-cadherin, vimentin, fibronectin and Slug, were reduced in OSC19 cells after treatment with GSPs in a dose-dependent manner (Figure 6B). Similar to GSPs, the treatment of OSC19 cells with erlotinib resulted in an increase in the levels of epithelial biomarkers (Figure 6C) and a decrease in the levels of mesenchymal biomarkers in OSC19 cells (Figure 6D).

**Figure 6:** Treatment of OSC19 cells with GSPs or erlotinib results in reversal of epithelial-to-mesenchymal transition. (**A**) Treatment of OSC19 cells with GSPs for 48 h enhanced the levels of epithelial biomarkers in the cells as assessed by western blotting, including the levels of E-cadherin, keratin-8, keratin-18 and desmoglein-2. (**B**) Simultaneously, the levels of mesenchymal biomarkers in cells, such as, N-cadherin, vimentin, fibronectin and Slug, were decreased in a dose-dependent manner. (**C and D**) Under identical conditions, treatment of OSC19 cells with erlotinib also resulted in reversal of epithelial-to-mesenchymal transition in a dose-dependent manner. Presented blots are representative of three independent experiments with similar results.

## Discussion

The therapeutic potential, including antitumor activity, of GSPs has been reported in various preclinical models [7]–[9], [22], [23]; however, the effect of GSPs on the invasive potential of cancer cells is less explored. In the current study, we investigated the potential utility of GSPs in the prevention of invasiveness of HNSCC cells. HNSCCs can arise from several different sub-sites. In our preliminary studies, we tested the invasiveness of HNSCC cell lines generated from the oral cavity, larynx, and pharynx. The results suggested that, under the experimental conditions used in these studies, these cell lines exhibited greater invasive potential than normal bronchial epithelial cells. The invasive potential of the metastatic OSC19 cell line that originated from the tongue was greater than the other cell lines (SCC1, SCC5, FaDu).

GSPs were found to inhibit the invasiveness of OSC19 cells in a dose-dependent manner and this inhibitory effect of GSPs was associated with the downregulation of EGFR expression in the OSC19 cells. The OSC19 cells overexpress EGFR and the inhibition of EGFR by GSPs may contribute to the inhibition of cell invasion of these cells. This concept is supported by the evidence that treatment of the OSC19 cells with gefitinib or erlotinib, small molecule inhibitors of EGFR, resulted in a reduction in the cell invasion ability. It has been reported that inhibitors of EGFR can prevent the growth and progression of HNSCCs; however, their long term use may also induce some form of toxicity [13]. Notably, significant toxicity has not been associated with the use of GSPs in animal models [7]–[9], [22].

NF-κB is a downstream target of EGFR, and activation of NF-κB has been identified as an important regulator of cancer cell invasion, metastasis and angiogenesis [14], [24], [25]. Therefore, we checked the effect of GSPs on the basal levels of NF-κB in OSC19 cells and found that treatment of these cells with GSPs results in downregulation as well as inactivation of the NF-κB pathway in a dose-dependent manner. GSPs decrease the levels of IKKα which is responsible for inactivation of NF-κB. Treatment of cells with caffeic acid phenethyl ester, an inhibitor of NF-κB, resulted in an inhibitory effect on the invasion of HNSCC cells. NF-κB-targeted proteins, such as MMPs, COX-2, iNOS and VEGF, have been implicated in tumor angiogenesis and tumor cell migration. Treatment of OSC19 cells with GSPs down-regulates the expression of these NF-κB-targeted proteins, which supports the evidence that NF-κB has a role in invasion of HNSCC cells, and that the inhibitory effect on cell invasion by GSPs is mediated, at least in part, through the inactivation of NF-κB. It is important to mention that all these effects of GSPs may not be solely caused by the inhibition of EGFR; other factors or targets may also play a role and that need to be identified. Proteins of the MAPK family are also downstream targets of EGFR and have been shown to play a crucial role in cancer cell migration/invasion. Activation of the proteins of MAPK family leads to the activation of NF-κB. Our results show that inhibition of invasiveness of OSC19 cells by GSPs is associated with the inhibition of ERK1/2 phosphorylation. The use of MEK inhibitor (UO126) blocked the cell invasion capacity of OSC19 cells, and this function of UO126 is similar to the action of GSPs. These observations suggest a possible involvement of the ERK1/2-NF-κB pathway in inhibition of the invasive potential of HNSCC cells by GSPs.

In addition to the role of NF-κB in cancer biology, such as in tissue invasion, cell migration and metastasis, NF-κB has been identified as an important regulator of EMT in several cancer cell types [14], [24], [25]. EMT plays a major role in invasion and metastasis of epithelial tumors. EMT can render tumor cells migratory and invasive through the involvement of all stages, invasion, intravasation and extravasation [16], [26]. During the EMT stage, cells change from an epithelial to a mesenchymal phenotype. They lose their characteristic epithelial traits and instead gain properties of mesenchymal cells. This process is coordinated primarily by the loss of epithelial biomarkers such as E-cadherin and certain cytokeratins, concomitant with the acquisition of mesenchymal markers, such as vimentin, fibronection, N-cadherin, *etc*.. In the present study, we found that GSPs treatment of OSC19 cells resulted in the suppression or loss of mesenchymal biomarkers while restoring the levels of epithelial biomarkers, which suggests that GSPs have the ability to reverse the EMT process in HNSCC cells. This may be one of the possible mechanisms through which GSPs reduce the invasiveness of HNSCC cells thereby inhibiting their invasion in our *in vitro* model.

Biological activity of phytochemicals largely depends on their bioavailability. The study of bioavailability and metabolism of any agent or phytochemical is an important part of all investigations. Some studies have been performed to examine the bioavailability and metabolism of proanthocyanidins. Studies have shown that polymeric proanthocyanidins are not absorbed as such in the gut [27]. The detection of proanthocyanidin dimers B1 and B2 in human plasma was reported in some studies [28], [29]. The absorption of these dimers was significantly lower than that of the monomeric flavanols [29]. However, these compounds were found to protect the intestinal mucosa against oxidative stress or the actions of carcinogens. Additionally, proanthocyanidins have been found to be quite stable, and GSPs are stable at least 2 years if stored in refrigerator at 4°C.

Together, the results from this study have identified for the first time that bioactive proanthocyanidins from grape seeds inhibit the invasiveness of human HNSCC cells and that this effect involves: (i) the inhibitory effect of GSPs on EGFR expression, (ii) the inhibitory effect of GSPs on the activation of the ERK1/2 proteins and inactivation of NF-κB, and (iii) reversal of the EMT. These events and observations are summarized in Figure 7. Further *in vitro* and *in vivo* studies may help to develop GSPs as a pharmacologically safe bioactive chemotherapeutic or chemopreventive agent when used either alone or in combination with other anti-metastatic drugs for the treatment of HNSCC in humans.

**Figure 7:** Summary of the action of GSPs on the prevention of HNSCC cell invasion. GSPs inhibit the expression levels of EGFR in human HNSCC cells, which plays a critical role in inactivation of ERK1/2, NF-κB and reversal of epithelial-to-mesenchymal transition. Collectively, these effects lead to GSPs-induced inhibition of cancer cell invasion. However, all these effects of GSPs may not be solely caused by the inhibition of EGFR expression; other targets may also play a role and that need to be further identified.
